# Dynamic Gesture Recognition Algorithm Based on 3D Convolutional Neural Network

**DOI:** 10.1155/2021/4828102

**Published:** 2021-08-16

**Authors:** Yuting Liu, Du Jiang, Haojie Duan, Ying Sun, Gongfa Li, Bo Tao, Juntong Yun, Ying Liu, Baojia Chen

**Affiliations:** ^1^Key Laboratory of Metallurgical Equipment and Control Technology of Ministry of Education, Wuhan University of Science and Technology, Wuhan 430081, China; ^2^Research Center for Biomimetic Robot and Intelligent Measurement and Control, Wuhan University of Science and Technology, Wuhan 430081, China; ^3^Hubei Key Laboratory of Mechanical Transmission and Manufacturing Engineering, Wuhan University of Science and Technology, Wuhan 430081, China; ^4^Hubei Key Laboratory of Hydroelectric Machinery Design & Maintenance, China Three Gorges University, Yichang 443002, China

## Abstract

Gesture recognition is one of the important ways of human-computer interaction, which is mainly detected by visual technology. The temporal and spatial features are extracted by convolution of the video containing gesture. However, compared with the convolution calculation of a single image, multiframe image of dynamic gestures has more computation, more complex feature extraction, and more network parameters, which affects the recognition efficiency and real-time performance of the model. To solve above problems, a dynamic gesture recognition model based on CBAM-C3D is proposed. Key frame extraction technology, multimodal joint training, and network optimization with BN layer are used for making the network performance better. The experiments show that the recognition accuracy of the proposed 3D convolutional neural network combined with attention mechanism reaches 72.4% on EgoGesture dataset, which is improved greatly compared with the current main dynamic gesture recognition methods, and the effectiveness of the proposed algorithm is verified.

## 1. Introduction

As a common means of communication in people's daily life, gestures also have great application in human-computer interaction. Compared with expressions, actions, and other interactive means, gestures are more intuitive, natural, and comfortable. Therefore, gesture communication is also the most used human-computer interaction means besides language [1, 2]. Gestures have a wide range of applications in human-computer interaction technology, such as intelligent driving, virtual reality, augmented reality [3, 4], medical assistance [5], and so on [6–8]. In intelligent driving, gestures are captured by vehicle intelligent control systems and analyzed by intelligent center. Instructions are sent out to complete the human control of vehicle navigation and entertainment functions [9, 10]. When talking about virtual reality and argument reality, Microsoft's HoloLens has already realized having entertainment of users in the virtual reality environment through both hands [11]. In medical assistances, gesture recognition can provide assistances for the hearing-impaired groups and realize the normal communication between deaf and dumb people.

Gestures could be mainly divided into dynamic and static. Static gestures focus on the hand posture and shape at a single point in time, such as gesture action “OK.” Only the spatial features of gestures are considered in recognition. Dynamic gesture recognition should not only consider hand postures and shapes but also pay attention to the spatial displacement and spatiotemporal correlation of the whole gesture [12–14]. Compared with static gesture recognition, dynamic gesture is closer to people's expression habits with more abundant information expression [15–17], which has more practical significance. Nowadays, researchers have proposed a variety of dynamic gesture recognition algorithms, including dynamic gesture feature extraction algorithm such as MEI algorithm, HOG algorithm, and HOF [18] algorithm and classification algorithm such as hidden Markov model [19]. With the development of deep learning, many video classification algorithms, for example, C3D [20] and dual stream convolution network and LSTM [21], have been applied to dynamic gesture recognition [22–24], achieving high recognition rate. However, the amount of network inputs is in large scale because of the need to extract the video spatial information and temporal information, which result in huge number of parameters and calculation. Such networks have complex network structure and low real-time performance. It is possible to increase the effect of dynamic gesture recognition by optimizing input and improving the existing feature extraction methods.

In this manuscript, we propose a dynamic gesture recognition algorithm based on attention mechanism of 3D convolutional neural network, which has several contributions:

- Interframe difference method is optimized. Input video data are processed to improve the problem of data redundancy and format inconsistency.
- 3D convolutional neural network is combined with attention mechanism. CBAM is used to optimize the structure of 3D convolutional neural network to reduce the transmission loss of input information and realize the feature extraction of spatial dimension and time dimension.
- Multimodal joint is applied to train neural network. To improve the effect of gesture recognition, the fusion method of dual-mode feature input is used to realize the feature complementarity of the two modes.

## 2. Related Work

As deep learning develops by leaps and bounds, computer vision has been promoted. Many excellent image analysis and recognition algorithms have been proposed. For example, the Alexnet which is designed by Srivastava [25] has achieved the best recognition performance in the Imagenet, an image recognition competition [26, 27]. Different from traditional methods of artificial design features, deep learning automatically extracts features through convolution neural network. By training and debugging the feature extraction network, more critical and representative spatiotemporal features can be extracted by deep learning for video classification and action recognition [28, 29]. The dynamic gesture recognition networks based on deep learning are mainly divided into three types: two-stream networks, long short-term memory (LSTM) network, and three-dimensional convolutional neural network (3D-CNN).

The concept of two-stream network was first proposed by Simonyan and Andrew [30] in 2014, and the optimal recognition effect was obtained in the behaviour recognition task of open data sets UCF-101 [31] and HMDB-5 [32]. The two-stream network algorithm also has some defects since the algorithm only gets spatial information through a single image. It is difficult to deal with the large changes in behaviour, and the optical flow image is only suitable for the small changes in motion information capture. Aiming at the problem of two-stream network, Wang et al. [33] designed a temporal segment network (TSN) to sparsely sample long time series images and obtain more robust spatiotemporal features through Inception v2 to improve the effect of action recognition. Based on the work of Wang et al., Feichtenhofer et al. [34] studied the method of fusing spatial and temporal information and found that the feature fusion in higher convolution layer of network has better recognition effect. In two-stream convolution networks, the operation of optical flow information could occupy a lot of memory and affect the recognition rate. Zhu et al. [35] designed a convolution network for optical flow estimation instead of optical flow information operation, cascaded temporal information network and spatial information network, and used multiple images stacked input to complete action recognition. Dynamic gesture recognition [36] is like action recognition. It also uses the algorithm to obtain the spatial and temporal information of the object expression in the video to realize the video action understanding.

LSTM is actually a type of recurrent neural network (RNN). Inputs of each layer of RNN consist of the output of the upper layer and the output of the same layer, and outputs of the neuron are the inputs of the same layer. Therefore, RNN could effectively deal with the problem of temporal feature extraction. However, the network can only solve the problem of short time series due to the limitation of structure. LSTM is designed to solve problem of long time series and historical information loss in the iteration. For the problem of information loss in long time sequence, LSTM controls the information processing of neurons with three structures: input gate layer, forget gate layer. and output gate layer. In the dynamic gesture recognition, LSTM uses the common convolutional network to extract the features, serializes the spatial features extracted by the previous network through LSTM, and then classifies them in the full connection layer.

3D-CNN is an improvement of convolution kernel and pooling method on traditional 2D convolution neural network. Continuous motions contain unique temporal information. However, 2D convolution kernel can only extract spatial information from image [37, 38], and 3D convolution kernel is designed to extract features from continuous image to obtain temporal information. Spatial scale pooling and channel scale pooling are also included in pooling process. Many scholars have studied 3D convolutional neural network. For example, Tran et al. [39] proposed C3D network to realize dynamic gesture recognition. The I3D network is proposed by Carreira and Zisserman [40]. Some previous excellent models are used in this algorithm. To solve the problem of excessive computing cost, Qiu et al. [41] proposed the P3D network, which optimized the convolution model.

Moreover, some algorithms use feature fusion to integrate image information and optical flow information, such as dual stream algorithm and MFFs-net algorithm [42]. The accuracy of the MFFs-net algorithm on Jester dataset is 96.28%, but the calculation of optical flow needs a lot of computing resources. Molchanov team has also done a lot of work in dynamic gesture recognition. In paper [25], the team proposed to integrate RGB image, depth image, and radar data to realize dynamic gesture recognition. In paper [43], the team proposed using 3D-CNN to train two different resolution networks and fusing the recognition results to improve the recognition accuracy. In paper [44], the team also used residual neural network to optimize 3D-CNN and verified the effectiveness of its model in SKIG data set and CharLearn2014 data set. Since the sign language data set also contains a large number of dynamic gestures, most dynamic gesture recognition models also use sign language as the data set for training and testing. In paper [45], a dual stream 3D-CNN is designed to realize dynamic gesture recognition based on effective fusion of multimodal data.

Based on the analysis of the above current research situation, it can be found that dynamic gesture recognition is still a research hotspot in the field of computer vision at present. Although it is still in the initial stage of this technology, the recognition of simple gesture has achieved good results in daily application. There are still some problems to be further studied and optimized.

## 3. 3D Convolutional Neural Network Based on Attention Mechanism

### 3.1. Structure of Dynamic Gesture Recognition Algorithm

Three aspects should be considered in motion recognition of video with single gesture:

- Appearance and texture feature of gestures
- Changes of gesture features, namely, gesture space features
- Time domain information between images, which is spatiotemporal characteristics of continuous changing gestures

In view of the above three aspects, this paper takes RGB image and depth image as input and designs a dynamic recognition model of three-dimensional convolutional neural network combined with convolutional block attention module (CBAM-C3D). The process (shown in Figure 1) is as follows: firstly, a key frame extraction method based on interframe difference method is designed to process the original input video. In this way, redundant frames of network input are reduced, and scale alignments of input data are realized. Then, the processed depth images and RGB images data are input into CBAM-C3D. Finally, the two data features are fused in series in the feature layer to complete the dynamic gesture recognition.

The proposed CBAM-C3D algorithm shown in Figure 2 is optimized according to the C3D network's structure which was proposed by Du et al. Batch normalization and ReLU layer are added into 3D convolution layer. The full connection layer and maximum pooling layer relate to CBAM network to optimize the features. This fusion network can not only reduce transmission loss of input information but also automatically learn important spatiotemporal information contained in images.

### 3.2. Key Frames Extraction of Dynamic Gesture

Due to the disunity of action standards and personal physical factors, the duration of the same action and gesture changes may be greatly different, which is also one of the difficulties of gesture recognition. There are two cases for the inconsistency of action duration:

- *Redundancy* of *Frames*. The input video sequences usually have many redundant frames without gesture action. These redundant images could greatly reduce the calculation speed of the network and even affect the recognition effect of the network.
- The time distribution of gesture movement is uneven. For complex gestures, it takes a long time to complete multiple gestures. In general, it cannot guarantee that the actions are carried out at a uniform speed, which makes the recognition process of dynamic gestures more difficult.

For these problems, the method of interframe difference to unify the scale of video data and simplify the data processing is proposed. The whole video is defined by several representative images.

The traditional inferframe difference method is mainly used for moving target monitoring. In this manuscript, it is optimized to obtain more accurate key frame images.  Figure 3 shows the calculation process of the inferframe difference method. Firstly, RGB-D image is used to segment the gesture area to obtain the hand image with the background removed. Then, the adjacent image pixel standard deviation algorithm is used to calculate the inferframe difference of the adjacent image in the image sequence. Finally, the size of the inferframe difference is sorted to complete the key frame extraction.

The standard deviation of inferframe difference *L*_*n*_ is the evaluation standard of key frames. For example, the number of key frames K is preset, and the standard deviation of the gray value change of the frame *n* image is calculated. The continuous images of the input video sequence are supposed to be *f*_*n*_ and *f*_*n*+1_. The pixels on images are (*x*, *y*). Gray values of the corresponding image are *f*_*n*_(*x*, *y*) and *f*_*n*+1_(*x*, *y*). According to formula (1), *f*_*n*_^*i*^ represents the gray value of pixel *i* of image *n*:

(1) $$\begin{array}{c} L\left(f_{n},f_{n+1}\right)=\sqrt{\sum_{i=1}^{n}{\left(f_{n}^{i}-f_{n+1}^{i}\right)}^{2}}. \end{array}$$

The maximum and minimum values of the sequence frame difference are counted, and intermediate value mid(*L*) is calculated according to formula (2). All local extremums less than mid(*L*) are removed and assumed that the number of remaining is *m*. Finally, the extracted extremum points are sorted, in which the frames corresponding to the first *K* extremum points are taken as the key frames. If *m* ≤ *K*, the last in the sequence is copied and filled based on *m* images.

(2) $$\begin{array}{c} \text{mid}\left(L\right)=\frac{\left(\max\left(L\right)+\min\left(L\right)\right)}{2}. \end{array}$$

### 3.3. Optimization of Three-Dimensional Convolutional Neural Network

#### 3.3.1. Optimization of Network Feature Extraction

Compared with SENet which only focuses on channel information extraction, CBAM considers the spatial information and channel information in feature extraction, that is, temporal features. In this paper, CBAM is used to optimize the structure of three-dimensional convolutional neural network, complete the important feature extraction of spatial dimension and time dimension, and strengthen the effect of network feature extraction.

(3) $$\begin{array}{c} I^{\prime }=A_{c}\left(I\right)⊗I,\\ I^{\prime \prime }=A_{s}\left(I^{\prime }\right)⊗I^{\prime }, \end{array}$$

where *I* ∈ *R*^*C*×*H*×*W*^ is feature map of input and *A*_*c*_ ∈ *R*^*C*×1×1^ and *A*_*s*_ ∈ *R*^1×*H*×*W*^ are one-dimensional and two-dimensional channel attention map, respectively.

Two vectors with only channel dimension are obtained by maximum pooling and average pooling in the spatial dimension. Then, the features are added and sigmoid activated by a two-layer neural network. The input of spatial attention processing can be obtained by multiplying the channel attention vector with the feature graph as follows:

(4) $$\begin{array}{c} A_{c}\left(I\right)=\sigma \left(\text{MLP}\left(\text{AvgPool}\left(I\right)\right)+\text{MLP}\left(\text{MaxPool}\left(I\right)\right)\right)\\ =\sigma \left(W_{1}\left(W_{0}\left(I_{\text{avg}}^{c}\right)\right)+W_{1}\left(W_{0}\left(I_{\max}^{c}\right)\right)\right), \end{array}$$

where *σ* is the sigmoid activation function. AvgPool()( ) and MaxPool()( ) represent average pooling and maximum, respectively. *W*_0_ ∈ *R*^*C*/*r*×*C*^ and *W*_1_ ∈ *R*^*C* × *C*/*r*^ are weights of MLP. This module is equivalent to a filter, the important channel weight is larger, and the unimportant channel weight is smaller. Therefore, it realizes the attention mechanism in the feature dimension.

To calculate spatial attention which concerns on the position of useful information, the maximum pooling and average pooling on the channel with only two channel dimensions are acquired. Then, the two vectors are input into a two-layer neural network, respectively. After feature addition, it is input into the convolution layer for weight optimization. In this way, a spatial attention filter is generated as follows:

(5) $$\begin{array}{c} A_{s}\left(I^{\prime }\right)=\sigma \left(f^{7\times 7}\left(\left[\text{AvgPool}\left(I\right);\text{MaxPool}\left(I\right)\right]\right)\right)\\ =\sigma \left(f^{7\times 7}\left(I_{\text{avg}}^{S};I_{\max}^{S}\right)\right), \end{array}$$

where *f* is the convolution operation.

The channel attention feature is input to the spatial attention mechanism network, and the spatial attention mechanism network is used to complete the feature extraction including space and temporal feature. Temporal attention concerns more on global information, while spatial attention focuses on local information. Therefore, the combination of these two attention modules will effectively extract salient features and enhance the expression of features.

#### 3.3.2. Optimization of Network Training Process

Due to the trend of polarization distribution and uneven distribution of data, gradient may disappear or explode. To solve this problem, BN layer is added to ensure the consistency of input data in each layer. The specific algorithm is as follows:

(6) $$\begin{array}{c} \mu_{\beta }=\frac{1}{n}\sum_{i=1}^{n}x_{i}, \end{array}$$

(7) $$\begin{array}{c} \sigma_{\beta }^{2}=\frac{1}{n}\sum_{i=1}^{n}{\left(x_{i}-\mu_{\beta }\right)}^{2}, \end{array}$$

(8) $$\begin{array}{c} {\hat{x}}_{i}=\frac{x_{i}-\mu_{\beta }}{\sqrt{\sigma_{\beta }^{2}+\varepsilon }}, \end{array}$$

(9) $$\begin{array}{c} y_{i}=\gamma {\hat{x}}_{i}+\beta . \end{array}$$

Formulas (6) and (7), respectively, calculate the mean value and variance of the data, formula (8) standardizes the data, and formula (9) offsets the data. After the data are processed by BN layer, the distribution of data will be more uniform, which is also conducive to improving the generalization performance of the network.

#### 3.3.3. Feature Fusion Strategy for Bimodal Data

In the field of behaviour recognition, many researchers have tried to use multimodal data as input to improve the recognition effect such as RGB image, depth image, and optical flow data. All kinds of modal data contain important information of gesture recognition, but the results of single-modal data recognition are not good enough. Therefore, the recognition efficiency of dynamic gesture is improved in this paper by fusing multiple modal data. Considering that 50 kinds of actions with significant difference in gesture are included, RGB images are used to fuse depth images for gesture recognition.

In this paper, RGB image and depth image are used as input data, and the two kinds of modal information are input into the CBAM-C3D model, respectively, by the way of training, and then the fusion is carried out after the respective features are obtained. Assume that the output feature vectors of the two kinds of modal information are *F*_RGB_ and *F*_Depth_, respectively, after feature extraction, and the final fusion feature vector is *F*_*u*_.

(a) Average fusion:
  (10) $$\begin{array}{c} F_{u}=\frac{1}{2}\left(F_{\text{RGB}}+F_{\text{Depth}}\right). \end{array}$$
(b) Series fusion:
  (11) $$\begin{array}{c} F_{u}=F_{\text{RGB}}⊗F_{\text{Depth}}, \end{array}$$
where ⊗ represents a tandem operation.

## 4. Experiment

### 4.1. Experimental Dataset

Different countries have different definitions of gesture, so there is no recognized dynamic gesture data set in this field. In order to facilitate multimodal data fusion training, this paper selects the EgoGesture [46] first person gesture database released by the State Key Laboratory of Pattern Recognition, Institute of Automation, Chinese Academy of Sciences in 2018 (Figure 4).

The dataset contains 2081 RGB-D videos, 24161 gesture samples, and 2953224 frames from six different themes. Each video sample is taken by Intel Realsense sr300 camera, and the data format is RGB-D. Each frame of video is 640 × 480 pixel resolution and 30 fps recording. There are 33 kinds of static and 50 kinds of dynamic gestures collected by 50 people from six different indoor and outdoor scenes.  Figure 5 is a schematic diagram of some gesture categories in EgoGesture database. As this paper mainly focuses on dynamic gesture recognition, we select 50 dynamic gestures and their labels as RGB data and depth data input to filter and adjust the EgoGesture database. Some samples of RGB and depth video data are taken as examples.

### 4.2. Experimental Environment and Training Parameters

All the experiments are carried out in Window10 system. The graphics card is NVIDIA gtx3060ti 8g. The running software environment is Python 3.6, Python-1.3.0 + torch vision-0.5.0, OpenCV-Python-4.5.0, and other auxiliary Python libraries. The data input is EgoGesture dataset, and the training set, test set, and verification set are divided according to the ratio of 3 : 1 : 1. When training the model, the model is verified and adjusted every 20 steps. Before network training, key frames are extracted from RGB images. RGB images and depth images are selected according to the number of frames. To increase the generalization of the model, the image is randomly clipped, and the initial input image of 240 *∗* 240 is randomly clipped to 112 *∗* 112. In the model training, the small batch stochastic gradient descent algorithm with momentum is used to optimize the 3D convolutional neural network. The number of training steps is 101, batch size is 16, initial learning rate is 0.01, and learning rate attenuation factor is 0.1 every 3000 iterations.

### 4.3. Comparison and Analysis

#### 4.3.1. Comparative Experiment of Different Inputs and Fusion Strategies

The single-mode input and dual-mode input are used for comparative experiments. RGB images, depth images, optical flow images, and RGB-depth images are selected to be input mode. Furthermore, average fusion and series fusion are used for dual-mode input in feature fusion layer. The input is 16-frame image set as input training, and the accuracy of the final dynamic gesture recognition result is shown in Figure 6.

Through the analysis of the experimental results, for the samples in the training set, in the use of the single-mode data input model, the recognition accuracy of RGB image is the highest, with a recognition accuracy of 52.5%. After fusing depth image input, the recognition accuracy is improved by 9.16%. It can be found that the multimodal data input model has better performance than the single-modal data input model. On the other hand, the multimode fusion input based on feature layer series connection has better effect, and the accuracy is 5.07% higher than the average fusion input. What can be inferred is that both input modes and fusion method influenced the performance of neural network. When the type of input data mode is fixed, using the appropriate data fusion method can make the characteristics of the object more prominent and train a better network performance.

#### 4.3.2. Comparative Experiment of Dual-Mode Data Fusion Strategy

For better reflecting the effectiveness of the multimodal feature fusion strategy, the confusion matrix is used to show effect of two different fusion methods. Figures 7 and 8 describe confusion matrices of two fusion methods of 50 kinds of gestures in EgoGesture dataset. The horizontal axis represents the categories predicted by the model for dynamic gestures, the vertical axis represents the real labels of dynamic gestures, and the right colour graph represents the prediction accuracy value and corresponding colour performance.

Comparing the two figures, it can be found that the average fusion model is easy to confuse some gesture recognition. For example, some confusions exist in gesture 1, 3, and 6 or gesture 2, 4, 5. These gestures do have similar features in motion trajectory and hand posture, which leads to misjudgment between them. After using the series fusion model, the false detection probability between these similar gestures decreases to a certain extent and the recognition accuracy is improved to a certain extent. Take gesture 2 as an example. In the average fusion confusion matrix, it can be found that the probability that gesture 4 is mistaken for gesture 2 is greater than 0.4 (the grid colour in the matrix can be compared with the colour bar on the right). However, in the series fusion mode, the probability that gesture 4 is mistaken for gesture 2 is less than 0.2. In general, the recognition effect and average recognition rate of the series fusion model are better than those of the average fusion model.

The above experiments show that in dynamic gesture recognition, the recognition model based on series fusion features can achieve better results mainly because it can save the features of each part when fusing. This method can avoid the loss of feature masking caused by direct fusion and can provide more complete feature information of the classifier so as to improve the performance of the whole model.

#### 4.3.3. Comparative Experiment of Key Frame Extraction

Most of the action frames range from 20 to 50, so 8 frames, 12 frames, 16 frames, and 20 frames are selected for experimental comparison. The interframe difference method optimized in this paper is compared with the traditional interframe difference method, and the advantages and disadvantages of the method are judged by accuracy, which is shown in Figure 9.

As can be seen from Figure 8, the accuracy of the optimization method in extracting 8, 12, 16, and 20 key frames is significantly improved compared with the traditional method, and the maximum recognition rate is increased by 2.82% from 60.45% to 63.27%. With the increase in the number of frames, the recognition effect is also improving. However, when the number of frames reaches 20, the recognition rate decreases. It is speculated that the number of frames of some gestures is less than 20. The key extraction process needs to expand the number, resulting in redundant frames, which will have a negative impact on the effect of gesture recognition.

#### 4.3.4. Overall Performance Evaluation of CBAM-C3D Model

The proposed dynamic gesture recognition method and other representative algorithms are tested on the EgoGesture dataset. The feasibility and effectiveness of this method are verified by comparative experiments. In Table 1, the accuracy of the proposed method is 72.4%, which is greatly improved compared with the traditional dynamic gesture recognition method.

## 5. Conclusions

A dynamic gesture recognition algorithm based on attention mechanism of 3D convolutional neural network is proposed in this manuscript. The optimized interframe difference method is used to deal with problems about video data redundancy and format disunity. Combined with CBAM network, the important spatiotemporal features are enhanced and invalid features are suppressed to realize the prominent expression of features. Finally, the dual-mode feature input fusion method is adopted to realize the complementary features of the two modes and improve the effect of gesture recognition. Meanwhile, the model designed in this paper is compared with other mainstream methods on EgoGesture dataset to verify the effectiveness of the proposed method. The recognition accuracy of the designed method is 72.4%, which is better than other networks.

This method also has some defects, such as large amount of network parameters and slow network prediction, resulting in poor real-time performance. It only recognized gesture for video containing a single action. Moreover, the dual-modal data fusion strategy proposed in this paper has mentioned that the input modal RGB image and depth image are related to each other, but this paper only fuses them on the feature layer. In the future work, it can be considered to fuse the dual-modal data in the preprocessing stage and increase the input modal information, such as the addition of optical flow data, to improve the recognition accuracy.

## Figures and Tables

**Figure 1:** The overall framework of the proposed algorithm.

**Figure 2:** Structure of the proposed CBAM-C3D networks. (a) is the connection methods. (b) is the structure of 3D-CBAM in the proposed networks.

**Figure 3:** Flow chart of the interframe difference method in video sequences.

**Figure 4:** Schematic diagram of some gesture categories in EgoGesture dataset.

**Figure 5:** Samples of RGB-D images: (a) scroll hand towards right; (b) scroll hand towards left.

**Figure 6:** Accuracy comparison of input data in different modes.

**Figure 7:** Confusion matrix of average fusion model.

**Figure 8:** Confusion matrix of series fusion model.

**Figure 9:** Comparison of accuracy of two key frame extraction methods.

**Table 1:** Results of different network models in EgoGesture.

Recognition methods	Input categories	Validation set of EgoGseture (%)	Test set of EgoGseture (%)
Harris3.5D	RGB + depth	35.8	36.1
HOG3D	RGB + depth	43.8	44.6
HON4D	Depth	57.2	58.3
C3D	RGB + depth	56.1	57.4
T3D	RGB + depth	62.4	63.8
R3D	RGB + depth	64.8	66.1
Proposed algorithm	RGB + depth	**71.5**	**72.4**

## Data Availability

The data used to support the findings of this study have not been made available because the relevant data involve legal issues and related confidentiality.
